The article "Ecopolitical discourse: Authoritarianism or democracy? — Evidence from China" was retracted in 2025. Reasons: unreliable results or conclusions; concerns about the peer review.

# Ecopolitical discourse: Authoritarianism or democracy? — Evidence from China

**DOI:** 10.1371/journal.pone.0239872

**Published:** 2020-10-01

**Authors:** Xinyun Hu, Mingming Li

**Affiliations:** 1 Research Centre of the Economy of the Upper Reaches of the Yangtze River, Chongqing Technology and Business University, Chongqing, China; 2 Department of Economics and Business, Central European University, Budapest, Hungary; University College London, UNITED KINGDOM

## Abstract

From the discourse analysis perspective, ecopolitics has experienced a discourse change from authoritarianism to democracy. This study uses theory of authoritarianism and democracy in ecopolitics to explore the impact of authoritarian ecopolitical discourse (AED) and democratic ecopolitical discourse (DED) on environmental quality in China. After analysis using panel data and comparison of three main regions, results suggest a negative relationship between AED of the central government and environmental quality. By contrast, a positive relationship exists between AED of local governments and environmental quality. A positive relationship exists between DED, which measures the proposals of People’s Congress deputies and Chinese People's Political Consultative Conference (CPPCC), and environmental quality. Nevertheless, the positive effect of DED is weaker than that of AED. The impact is also different among the regions. Our interpretations are as follows. China’s current governance mechanism is a top–down decision-making mechanism, rather than a bottom–up information transmission mechanism. The concentration of power keeps decision-making power and resources away from levels with considerably accurate information and capabilities in problem solving. Therefore, we suggest that governments should change their decision-making process and exert effort to be transparent to the entire society. A bottom–up mechanism of information collection and transmission should be established, such as environmental inspection mechanism and checking on cadres’ achievements with green GDP.

## 1 Introduction

Ecological problems lie between the natural and social systems, and the alleviation of ecological crisis inevitably points to the innovation of political thinking. As a political animal, people’s social practice cannot be separated from the related field of natural environment, thereby indicating a natural connection between ecological environment and politics [1]. Therefore, ecological politics (or ecopolitics) has gradually developed into a global political issue of universal significance. Ecopolitics is a political ideology that aims to foster an ecological and sustainable society rooted in nonviolence, environmentalism, social justice, and grassroots democracy [2]. The essence of ecopolitics is to raise the issue of eco-environment to a political level, thereby integrating the development of politics and eco-environment and ultimately promoting the sustainable, healthy, and stable development of global politics and eco-environment [3]. Since the 1980s, the deteriorating environment of the earth has posed a serious threat to human survival and development. “Ecological participation in politics” has been placed on the agenda of politicians in developed countries. They know that only by focusing on ecological protection can they win the support of voters and the trust of Parliament. They used the enthusiasm of young environmentalists to form political groups and intervene in state affairs. Simultaneously, international organizations, such as the United Nations Environment Program, have also integrated ecological issues into international political affairs.

Ecopolitics has long been accused of authoritarian tendencies in its development. However, the authoritarianism of environmental governance has its supporters in theory and practice. On the one hand, the professionalism and complexity of environmental problems urgently require the government to use rapid and efficient authoritative means of governance [4]. On the other hand, the unity and compulsion of authoritarianism are conducive to solving environmental problems immediately and effectively [5]. However, the emphasis of environmental authoritarianism on governmental governance and regulatory means will inevitably lead to the lack of effectiveness of environmental governance and difficulty in achieving the rationality of environmental value [6]. By contrast, the participation, openness, and prudence of environmental democracy are internally compatible with the publicity and complexity of environmental problems, which can compensate for the deficiency of environmental authoritarianism [7]. Note that environmental democracy still needs government participation. Such a participation is the correction and remedy of the government’s environmental administrative crisis.

With the escalation of contradiction between economic growth and environmental quality, China as a developing country has also placed “ecopolitical participation” on the agenda of governments with the pace of developed countries. On January 4, 2016, the central environmental protection supervision group, which is known as “environmental protection envoy,” was officially established. Accordingly, Hebei was selected as the first station for supervision. The central environmental protection supervision group is led by the Ministry of Environmental Protection, with the participation of relevant leaders of the Central Commission for Discipline Inspection and Central Organization Department, and carries out environmental protection supervision on behalf of the Party Central Committee and State Council. As of August 15, 2019, eight central environmental protection supervision groups have completed the supervision of six provinces and two central enterprises. The supervision teams accepted 18732 public tip-offs. The protection of ecological environment has become the crucial strategic goal of governments. However, the authority of the government does not seem to be enough to change the current situation of environmental pollution in China. China's one-dimensional incentive mode with GDP as the core has led to obvious distortion of local government motivation. In the case of fiscal decentralization accompanied by political centralization, local government officials sacrifice environment to promote economic growth in order to obtain political promotion [8]. Different interest demands of the local and central governments, as well as the competition among the local governments, have induced and intensified regional environmental interest conflicts [9]. The evident paradox within China’s environmental politics is the huge gap between the central government’s policy and its implementation outcomes at the local levels.

In addition to the above-mentioned top-down pressure, are there other forces or factors that will promote environmental governance? The existing ecological politics has experienced the tendency from authoritarianism to democracy [10]. From the experience of developed countries, the initial impetus of environmental protection comes from the public, such as the emergence of foreign green party [11–13]. In China, with the continuous improvement of urban residents' attention to the quality of life and the enhancement of environmental information transparency, especially the development of modern media, more and more people begin to express their concern about pollution and their strong demand for environmental governance consciously and systematically. However, the development of environmental democracy in China is only the tip of the iceberg. Many environmental mass incidents may have been suppressed in the early stage, and the public's voice has not been met. Although this bottom-up mechanism is effective in foreign countries, whether it is equally effective in China is a matter of great concern to both academic and decision-making circles.

To sum up, under the current social and institutional environment in China, the impact of environmental authoritarianism and environmental democracy on China's environmental governance requires further study. To explore this issue, the remainder of this paper is organized as follows. Section 2 presents a theoretical review of authoritarianism and democracy in ecological politics, and proposes relevant theoretical hypotheses. Section 3 introduces the measurement of authoritarian ecopolitical discourse (AED) and democratic ecopolitical discourse (DED). Section 4 uses the technique for order preference by similarity to ideal solution (TOPSIS) method to calculate a comprehensive evaluation index system of China’s environmental quality. Section 5 applies the empirical study regression to maximize the relationship between authoritarian/democratic ecopolitical discourse and environmental quality in China, particularly by using the fixed effect–instrumental variables method to perform the analysis of regional difference, thereby further verifying the hypotheses. Section 6 presents the conclusion, suggestion, and future directions.

## 2. Literature review

### 2.1. Concepts and definitions

The essence of ecopolitics is the product of discourse practice, and it emerges, evolves, and develops in discourse practice. Ecopolitics, as a combination of theory and practice to understand the relationship between ecology and politics, is a form of epistemology [14]. Accordingly, this concept can explain the knowledge world of interaction between ecology and politics through discourse evolution and analysis. The appearance and development of ecological politics process contains extensive dialogue, rhetoric, and symbolic elements or debate “discourse”; thus, discourse reflects the knowledge of ecopolitics [15]. With the help of the discourse medium, people constantly provide new ideas to the social background through the expression of “significance.” Subjective construction (cognition) must be realized through linguistic symbols. However, discourse is not without foundation but generated under a complex social interaction and cultural background, which is called context [16]. The ecopolitical discourse is mainly constructed through four dimensions, namely, views on ecology, decision-maker of the generation of knowledge, rules of discourse formation and the way to objectify knowledge. The ecopolitical discourse has experienced the transformation from authoritarianism to democracy, which mainly reflected in the changes of these four dimensions [17], shown in Table 1. In general, the idea of using political thinking to alleviate ecological crisis can be relatively summarized in two consecutive and opposite discourse systems, namely, authoritarian ecopolitical discourse (AED) and democratic ecopolitical discourse (DED).

**Table 1:** Framework of the authoritarian & democratic ecopolitical discourse.

	Authoritarian	Democratic
Views on ecology	Nature is subordinate to human society; the social and political pattern of "center-edge"	Equality of human, nature social problems; fairness and justice; competition and cooperation
Decision-maker of the generation of knowledge	Administrative state; technical bureaucrat; expert	Citizens; stakeholders
Rules of discourse formation	Technical narratives	Networking narratives
The way to objectify knowledge	Public interest under technical narratives; authority's discourse right	Expectations for consensus; acknowledge the existence of difference

### 2.2. AED

Authoritarianism holds that ecological crisis should be alleviated by the high efficiency of state administration. The early ecopolitical thinking focused on the significance of authoritarianism to the alleviation of ecological crisis. In the eyes of supporters of limited resources theory, the environment exists as a type of “resource” and has substantial economic significance [18]. Heilbroner stated that we could avoid the internal contradictions and serious social polarization caused by resource competition only through large-scale state management and coercive power [19]. Authoritarian discourse doubts whether free market itself can achieve ecological security. Private economic activities and completely market-based distribution mechanism have become the institutional root of environmental pollution and ecological damage [20]. The urgency of ecological crisis requires a repressive centralized government to formulate environmental rules, allocate resources, and control population. To avoid ecological crisis, we need to transfer the right to the elite at the expense of people’s interests [21]. Paehlke believed that democratic politics and economic structure cannot cope with ecological crisis, and tended to choose a “brave new world.” What the world implements is a set of authoritarian system, which takes a relatively kind attitude toward ecology [22]. In many cases, the low efficiency of democracy and its limitation in coordinating different interests affect the improvement of governance performance [23]. Accordingly, ecological crisis can be effectively controlled with a strong centralized bureaucracy and advanced technology [24]. AED regards the administrative state as the leading mechanism to alleviate ecological crisis, and the administrative state and technical bureaucrats determine the formation of ecopolitics, as shown in Table 1. China is an authoritarian country and adopts political centralization. In China’s political centralization, knowledge generation is mainly decided by the central government, which we can regard as part of authoritarianism. According to the above analysis, we propose the following hypothesis:

Hypothesis 1 (H1): *A positive relationship exists between AED of the central government and environmental quality of China*.

Political centralization of China means that the upper government has stronger power to appoint and remove lower government officials [25]. Therefore, the upper government can guarantee that its behaviors and values are the same with the lower government in a macro direction. This system rebuilds the incentive mechanisms of local governments and leads their value orientation, thereby forming a system represented by pressure [26, 27]. Given the Chinese political centralization and its resulting GDP championship and campaign-style environmental inspection, the central government’s environmental governance intentions were passed on to the provincial governments, which are the real executors to solve environmental problems [28]. China’s current environmental governance mechanism is a top–down decision-making and implementation mechanism [29]. The actual operators of environmental governance are local governments, which obey the orders of the central government [30]. In other words, local governments are also the specific manifestations of authoritarianism and can influence the environmental level. According to the theory of environmental authoritarianism mentioned above, the high efficiency of State Administration has a positive impact on environmental governance. Thus, we propose the following hypothesis:

Hypothesis 2 (H2): *A positive relationship exists between the AED of the local governments and environmental quality of China*.

However, the possibility exists of mutual influence between the central government and local governments. Given that this phenomenon will eventually affect the regression result, we will choose the appropriate instrument variable method in the panel data for the central government ecopolitical discourse to solve this problem in Section 5.

### 2.3. DED

In the face of the trend that ecological politics is likely to slide to authoritarianism, democracy places the right to use discourse on the disclosure of power relations and ideology behind authoritarianism. Saward believed that democracy should include environmental concerns if we want to protect the basic democratic rights of citizens, because citizens have the right to be free from certain preventable environmental risks [10]. Hence, democrats must be environmentalists. Dobson proposed the ecological citizenship right when he discussed how to overcome the inconsistency between individual behavior and individual attitude based on sustainable development goals [31]. Some scholars who support environmental democracy strongly oppose environmental authoritarianism. For example, Escobar expressed that “sustainable development,” as a type of discourse, is a cover up of power relations and has “the potential intention to promote the capitalization of the natural environment [32].” In the view of democratic pragmatists, complex ecopolitical knowledge cannot be controlled by authoritative institutions because these institutions and experts, who master scientific and technological discourse, are given power, thereby forming a “power domination” of ecopolitical knowledge [33]. Since the 1960s, Japanese citizens have launched large-scale legal proceedings, and the media have also tracked and reported pollution accidents. Non-governmental organizations against environmental pollution have also been set up in many areas. In the 1970s, the American “Not in my Back Yard,” an environmental public consultation and environmental right to know legislation, developed correspondingly, thereby manifesting democratic ecopolitics. At the same time, the green party has started to spread in Europe and various kinds of non-governmental organizations of environmental protection have emerged in succession. The voice of environmental democracy is gradually rising. In general, DED regards citizens and their stakeholders as participants and decision makers of ecopolitical knowledge, and regards the relationship between ecology and politics as an equal political interaction of multiple subjects, also shown in Table 1.

Although China emphasizes centralization, it also tends to multi-agent environmental governance [34–36]. In China, a growing number of people has expressed their concerns about pollution and strong demands for environmental governance. These appeals affect the government's decision and have a positive impact on environmental governance. For example, in July 2012, people in Shifang held a demonstration to protest against the construction of molybdenum copper project and then the project was put on hold. At the end of the same month, group unexpected incidents to boycott the waste water discharge project of paper mills broke out in Qidong City. Facing strong appeals from the public, the government decided to cancel the project. Although these mass incidents have achieved some progress and foreign environmental democracy has also made us optimistic about the role of public appeals, the success of these public wishes is only the tip of the iceberg compared with hundreds of environmental pollution incidents in China. Some special cases of large-scale environmental events may have "selective bias", which may not represent the general and common situation. Besides, the current governance mechanism in China is still a top-down environmental governance structure rather than a bottom–up information collection and transmission mechanism. Therefore, it can be seen that environmental democracy has a positive effect on the improvement of China's environment, but its effect is limited and may be weaker than that of environmental authoritarianism in China. Thus, we propose the following hypothesis:

Hypothesis 3 (H3): *A positive relationship exists between DED from people’s appeal and environmental quality*. *However*, *the positive effect is lower than that of AED*.

## 3 Measuring AED and DED

### 3.1 Measuring AED and DED

As mentioned in Section 2, ecological politics is mainly divided into two consecutive and opposite discourse systems, namely AED and DED. The ecopolitical discourse is mainly constructed through four dimensions and the transformation of the discourse from authoritarianism to democracy is mainly reflected in the four dimensions, especially the second one, which reflects the process of the gradual dissolution of subject's centrality.

Discourse is the language that the subject speaks or writes. Discourse analysis refers to the study of the social consequences brought by subject's narration and the way of narration [31, 32]. Foucault’ s discourse analysis is the specific language patterns intertwined with social power and an activity between the speaker and the receiver through text or communication in a specific social context [37]. This shows that discourse can be reflected in the text, representing the attention of knowledge producers to a certain field of society in the process of communication. Some studies have shown that attention can affect decision-makers' behavior and decision-making effect. Dahl and Simon believed that the key to decision-making is how decision-makers effectively allocate their limited attention [38]. Ocasio held that decision-making depends on attention-focused issues [39]. Stone et al. introduced attention study into the field of government management, explored the factors affecting the conversion of government policy decisions, and proposed an "attention-driven policy choice model". The model shows that the choice of government behavior mainly depends on the factors that most attract the government's attention [40]. In this paper, environmental governance is a common behavior choice of governments and the public. The two opposite discourse systems, AED and DED, reflect attention of governments and the public to ecological environment, and then affect the behavior and effect of decision-makers on environmental governance.

Measuring AED and DED needs to find a reliable text that can scientifically reflect the ecopolitical discourse of environmental authoritarianism and environmental democracy. This paper tries to use text extraction to measure AED and DED to reflect governments and the public's attention to the environment. Some scholars have used text extraction to explore urban environmental governance, such as using Google Trends and Google search to construct indicators to measure the public's attention to environmental issues [41, 42]. Based on China's special situation, this paper chooses two kinds of documents that are highly related to China's ecological authority and ecological democracy, namely central/local government work reports and proposals of the People's Congress and the Chinese People's Political Consultative Conference (CPPCC).

The reason why the central and local government work reports can be used as authoritarianism discourse is that Chinese governments prefer command-and-control governance. This type of governance is related to the operating mechanism of the administrative system of socialism with Chinese characteristics that emphasizes centralization. Correspondingly, Chinese government work reports are official documents with statutory effects and policy texts issued during the two sessions with the nature of the policy agenda [43]. As the official expression of government intention on management, these reports have a standardized writing style and rigorously use vocabulary and syntax. They are also the baton for the government to allocate resources and devote energy, and have immense practical and instructive significance for the relevant personnel to immediately understand domain knowledge. This study uses word frequency statistics to selects keywords related to ecological environment in government work reports. Because frequently used words that are the center of subject’s cognition can reflect its cognitive tendency and the most active part of their thinking [44]. Word frequency is an extremely important variable in researches on word processing and memory [45]. The use of statistical technology of word frequency to extract text information to quantify AED is an important contribution of the current study, and is different from the existing literature.

The reason why the proposals of People’s Congress deputies and CPPCC can be used as democracy discourse is that they are important parts of the implementation of socialist democracy. Both People’s Congress deputies and CPPCC have the power to propose proposals and are channels for the public to speak out. They can supervise governments and put pressure on them. On the one hand, the suggestions put forward by deputies to the people's Congress are an important form for the people to exercise their democratic power and participate in the management of state affairs. Deputies to the people's Congress involving people at the grass-roots level are elected by the people, so they are more representative of the people's power and their suggestions are closely related to the vital interests of the general public. On the other hand, CPPCC plays its role in political consultation, democratic supervision and participation in and deliberation of state affairs and the CPPCC's proposals are put forward by the democratic parties, social organizations and members of the CPPCC to the plenary session or standing committee of the CPPCC and they are manifestation of socialist democracy. Therefore, this paper uses the ratio of the number of proposals about ecological environment of People’s Congress and Chinese People’s Political Consultative Conference (CPPCC) in 10,000 people to quantify DED is an important contribution of the current study.

### 3.2 Logic of word frequency statistics

We collect local government work reports from 29 provinces (excluding Hainan and Xizang provinces due to lack of data; 319 copies) and central government work reports (11 copies) from 2004 to 2014 (330 copies). Information is extrapolated from the State Council’s Work Reports [46] and Documents of Provincial Governments [47].

First, 330 government work reports are merged. The R language “Jieba” (Chinese for “to stutter”) Chinese word segmentation module [48] is used to segment the text automatically. “Jieba” Chinese text segmentation is one of the important tools for text mining and built to be the best Python Chinese word segmentation module. Second, this study combines the connotation of word frequency with the research dimension of ecological environment according to the ranking of the number of word frequency. Furthermore, this research individually and manually selects key words about ecological environment. Given that low-frequency words often fail to show sufficient attention, only the key words with frequency of no less than 10 are included in the “word bag,” thereby ensuring that the selected key words can reflect the research emphasis. Third, the key words are confirmed in the specific context to solve the inconsistency of lexical meaning, thereby ultimately obtaining the key words (Parts are shown in S1 Appendix). Lastly, total number of keywords, number of sentences containing keywords (NSK), and total number of sentences (TNS) reflecting the ecological environment are calculated.

The frequency of a word in the text also depends on the length of the text. The frequency of a word in a long text is more, whereas that in a short text is less; thus, the information quantity of the latter can never be considered larger than that of the former [49]. The key words need to be further standardized to increase robustness and solve the problem of incomparable results owing to the different length of information text. Based on the preceding analysis, AED is represented by the ratio of the number of sentences containing key words and total number of sentences. The formula is as follows:

AED=NSK/TNS (1)

This study separates AED for the central government from 29 local governments. The AED of the central government (CAED) comes from information extraction of central government reports, whereas the AED of local governments (LAED) is abstracted from the information from the local government reports.

## 4 Measuring environmental quality of China

The ecological environment is a complex system that cannot be measured by a single variable. Therefore, we need to build an index system with multiple variables to calculate the comprehensive assessment value of environmental quality using the comprehensive index evaluation method. With the deep understanding of things, the evaluation of things is often a comprehensive judgment under the interaction of multiple factors. The comprehensive evaluation model refers to an entire comprehensive evaluation value synthesized using multiple evaluation index values through a certain mathematical model. This model’s advantages lie in comprehensiveness (including multiple indexes, thereby reflecting the multiple aspects of things), integrity (making overall judgment on the evaluated object), and generality (explaining the general level of the evaluated object with a comprehensive index).

We establish a comprehensive evaluation index system of China’s ecological environment with 19 indexes (*x*_*1*_*–x*_*19*_,), as shown in S2 Appendix. Data used in this section is taken from the *China Environmental Statistics Yearbook*, *China Environmental Yearbook*, and *China Statistical Yearbook* (also see S2 Appendix). We comprehensively evaluate the environmental quality using the TOPSIS method. The detailed processes are presented in the following subsection.

First, Eq (2) is used to normalize the original data *x*_*ij*_ (i is region and j is index) to eliminate the dimension and obtain the analysis data matrix in Eq (3).

$$z_{ij}=x_{ij}^{}/\sqrt{\sum_{i}x_{ij}^{2}}$$ (2)

$$z=\left[\begin{array}{cccc} z_{11} & z_{12} & \cdots & z_{1p}\\ z_{21} & z_{22} & \cdots & z_{2p}\\ \cdots & \cdots & \cdots & \cdots \\ z_{n1} & z_{n2} & \cdots & z_{np} \end{array}\right]$$ (3)

Second, we determine the optimal and worst values of each index, and establish the best value vector z^+^ in Eq (4) and worst value vector z^-^ in Eq (5).

$$z^{+}=\max_{n,j}\left(z_{1}^{+},z_{2}^{+},\ldots ,z_{p}^{+}\right)$$ (4)

$$z^{-}=\min_{n,j}\left(z_{1}^{-},z_{2}^{-},\ldots ,z_{p}^{-}\right)$$ (5)

Third, we calculate the distance between each evaluation object and the optimal value in Eq (6), and the distance between the evaluation object and worst value in Eq (7).

$$D_{i}^{+}=\sqrt{\sum_{j}{\left(z_{ij}-z_{j}^{+}\right)}^{2}}$$ (6)

$$D_{i}^{-}=\sqrt{\sum_{j}{\left(z_{ij}-z_{j}^{-}\right)}^{2}}$$ (7)

Eq (8) is used to calculate the relative proximity between each evaluation index and the optimal value:

$$C_{i}=\frac{D_{i}^{-}}{D_{i}^{+}+D_{i}^{-}}$$ (8)

Lastly, *C*_*i*_ is the environmental quality of different regions *i* in a certain year. The preceding steps are used to calculate the environmental quality of different provinces *i* in different years *t* called *C*_*it*_ (i.e., 29 provinces from 2004 to 2014 in this study).

## 5 Estimating equations and empirical results

### 5.1 Data sources and descriptive statistics

#### 5.1.1 Description of environmental quality

Our analysis is performed using the data of the entire provinces in Mainland China (excluding Hainan and Xizang provinces due to the limitation of data, 29 provinces totally) between 2004 and 2014. According to the national real estate development investment and sales of 2016 released by the Bureau of Statistics in January 2017, we divide the entire China into three main regions: Eastern, Middle, and Western regions. The Eastern region includes Beijing, Tianjin, Hebei, Liaoning, Shanghai, Jiangsu, Zhejiang, Fujian, Shandong, and Guangdong. The Middle region includes Shanxi, Jilin, Heilongjiang, Anhui, Jiangxi, Henan, Hubei, Hunan, Inner Mongolia, and Guangxi. The Western region includes Chongqing, Sichuan, Guizhou, Yunnan, Shaanxi, Gansu, Qinghai, Ningxia, and Xinjiang. The data of environmental quality of China (C) as a dependent variable is taken from the calculation of comprehensive index in Section 4. Figs 1–4 present a detailed illustration of C of the entire country and the three regions. From a macro perspective, the quality is improving but continues to be different among the regions and even the provinces within a single region.

**Fig 1:** Environment quality (C) of China.

**Fig 2:** Environment quality (C) of West Region.

**Fig 3:** Environment quality (C) of Middle Region.

**Fig 4:** Environment quality (C) of East Region.

#### 5.1.2 Description of the explanatory variables

The CAED and LAED data reflecting AED is taken from the extraction of word frequency of the central and local government work reports from 29 provinces from 2004 to 2014 (in Section 3.2). The report with the fewest words includes over 10000 Chinese characters, whereas the one with the most words includes 32,000 Chinese characters. The average number of words per annual work report is 17,000 Chinese characters. The Table 2 shows the AED for both central and local government.

**Table 2:** (a) AED for the central government (CAED). (b) AED for the local government (LAED, Part).

Year	TNS		NSK	CAED
2004	519		47	9.06%
2005	625		67	10.72%
2006	636		77	12.11%
2007	603		108	17.91%
2008	762		114	14.96%
2009	609		82	13.46%
2010	608		84	13.82%
2011	590		86	14.58%
2012	558		86	15.41%
2013	372		51	13.71%
2014	512		82	16.02%
Year	Province	TNS	NSK	LAED
2004	Anhui	370	50	13.51%
2005	Anhui	338	42	12.43%
2006	Anhui	318	61	19.18%
2007	Anhui	267	58	21.72%
2008	Anhui	480	107	22.29%
2009	Anhui	396	81	20.45%
2010	Anhui	475	90	18.95%
2011	Anhui	530	112	21.13%
2012	Anhui	399	71	17.79%
2013	Anhui	412	77	18.69%
2014	Anhui	343	75	21.87%

DED represents people’s environment appeal that is expressed by the ratio of the number of proposals about ecological environment of People’s Congress and CPPCC in 10,000 people. Other control variables that may affect the comprehensive level of China’s ecological environment are GDP per capita (PCGDP), industrial structure (IS), energy efficiency (EF), and energy structure (ES). The data of control variables were taken from the *China Environmental Statistics Yearbook*, *China Environmental Yearbook*, and *China Statistical Yearbook*.

Table 3 shows the observation of the variables, means, standard deviations, and related index of data. The fiscal investment of local governments in environmental governance (LFI) of the 29 provinces from 2004 to 2014 will be used as instrumental variable in Section 5.2.2. These data are also listed in Table 3 and will be discussed further in the succeeding sections. The LFI data were sourced from the *China Statistics Yearbook*.

**Table 3:** Descriptive statistics.

	N	Mean	St.Dev	p1	p99	t-value
C	319	.32	.14	.06	.68	42.16
LAED	319	.021	.006	.01	.03	65.33
CAED	11	.14	.02	.09	.18	18.46
DED	319	.46	.31	0	1	26
PCGDP	319	17190.29	10847.78	4975.74	52807.05	28.3
ES	319	2.16	1.01	.83	5.13	38.37
EF	319	98.44	35.28	33.82	199.17	49.83
IS	319	2.26	.13	1.91	2.75	301.9
LFI	319	193.96	192.6	12.69	980	17.99

### 5.2 Empirical model

Our empirical analysis has two main targets. First, we need to exploit the influence of AED and DED on environmental quality in China, and distinguish the central from local governments. Second, the comparison among the aforementioned regions has a significant meaning for practical environment policy-making and execution. The following basic empirical model (9) is established based on data in Section 5.1 after logarithmic processing, where *X*_*it*_ are the control variables, including *LnPCGDP*_*it*_, *LnIS*_*it*_, *LnEF*_*it*_, and *LnES*_*it*_; and region is the dummy variable.

$$\begin{array}{l} {\mathrm{LnC}}_{\mathrm{it}}=\alpha_{\mathrm{it}}+\beta_{1}{\mathrm{LnCAED}}_{t}+\beta_{2}{\mathrm{LnLAED}}_{t}+\beta_{3}{\mathrm{LnDED}}_{\mathrm{it}}\\ +\beta_{4}*region+\beta_{5}*region*LnPCGDP_{it}+\beta *X_{it}+\varepsilon_{it} \end{array}$$ (9)

#### 5.2.1 Pooled regression

First, we use the pooled ordinary least squares (OLS) regression for the rough analysis. Eq (9) can be specifically written as follows:

$$\begin{array}{l} LnC_{it}=\alpha +\beta_{1}LnLAED_{it}+\beta_{2}LnCAED_{t}+\beta_{3}LnDED_{it}+\beta_{4}Middle_{it}\\ +\beta_{5}Westit+\beta_{6}*Middle_{it}*LnPCGDP_{it}+\beta_{7}*West_{it}*LnPCGDP_{it}\\ +\beta_{8}LnPCGDP_{it}+\beta_{9}LnISit+\beta_{10}LnEF_{it}+\beta_{11}LnES_{it}+\varepsilon_{it} \end{array}$$ (10)

Table 4 presents the pooled regression results of Eq (10), which shows that AED of the central government has a negative correlation with environmental quality, with a significance level of at least 1%. This result indicates that the strengthening of the central government’s authoritarianism has a negative impact on the environment. From the coefficient value perspective, a 1% increase in AED of the central government will cause a 0.05% decrease in environmental quality. This result is in contrast with H1, which states that a positive relationship exists between the AED of the central government and environmental quality of China.

**Table 4:** Regression results of the pooled regression.

	(1)	(2)	(3)	(4)
VARIABLES	lnC	lnC	lnC	lnC
lnCAED	-0.109	-0.107	-0.118	-0.0443
	(0.110)	(0.112)	(0.105)	(0.0899)
lnLAED	0.102	0.103	0.147	0.156*
	(0.116)	(0.116)	(0.109)	(0.0934)
lnDED	0.0175	0.0176	0.00598	0.0438***
	(0.0186)	(0.0187)	(0.0176)	(0.0155)
Middle	-4.726*	-4.699*	-1.588	-9.752***
	(2.454)	(2.484)	(2.374)	(2.172)
West	-7.524***	-7.485***	-4.030**	-8.193***
	(1.473)	(1.569)	(1.559)	(1.391)
Middle*lnPCGDP	0.426	0.424	0.0949	0.958***
	(0.259)	(0.262)	(0.250)	(0.229)
West* lnPCGDP	0.711***	0.707***	0.347**	0.817***
	(0.153)	(0.163)	(0.162)	(0.146)
lnPCGDP	-0.451***	-0.446***	-0.191	-0.445***
	(0.0979)	(0.117)	(0.117)	(0.103)
lnIS		-0.0421	0.306	0.953**
		(0.572)	(0.538)	(0.465)
lnEF			0.498***	0.784***
			(0.0750)	(0.0696)
lnES				-0.750***
				(0.0704)
Constant	3.615***	3.609***	-1.314	0.111
	(1.132)	(1.136)	(1.298)	(1.119)
Observations	319	319	319	319
R-squared	0.291	0.291	0.380	0.547

Note: The values in parentheses are standard errors;

*** represents p <0.01,

** represents p <0.05, and

* represents p <0.1.

For H2, Table 4 shows that AED of local governments is significantly positively related to environmental quality, thereby indicating that the strengthening of their authoritarianism positively impacts environmental quality. The results of the general pooled regression indicate that the coefficients of LAED are approximately 0.259. That is, when AED of local governments increases by 1%, environmental quality improves by 0.15%. This result is consistent with H2, which states that a positive relationship exists between AED of the local governments and environmental quality of China.

For H3, Table 4 shows that DED is significantly positively related to environmental quality, thereby indicating that people’s appeal for ecological environment play an important role in improving environmental quality. The results of the general pooled regression indicate that the DED coefficient is approximately 0.044. That is, when people’s appeal for ecological environment increases by 1%, environmental quality improves by 0.0444%. However, the effect of DED is evidently weaker than that of AED of local governments. This result is consistent with H3, which states that a positive relationship exists between the DED from people’s appeal and the environmental quality of China.

The analysis of the other coefficients is as follows. The coefficient of the dummy variables of the other regions are compared with those of the Eastern region. In particular, −9.752 in column 4 indicates that environmental quality in the Middle region is considerably worse than that in the Eastern region. Similarly, −8.193 indicates that environmental quality in the Western region is also substantially worse than that in the Eastern region. We can explain that the economy in the East is significantly developed, thereby prompting governments to considerably focus on environmental governance in this region. Moreover, the coefficients of the cross-term between per capita GDP and regions show that the Western and Middle regions are committed to improving GDP, which has a positive and significant effect on environmental quality.

When the control variables are considered, 1% increase in GDP leads to 0.445% decline in environmental quality, thereby indicating that an increase in GDP per capita does not mean an increase in environmental quality. This finding fits the conventional conception. China’s economic development has been at the expense of environmental quality in the past 10 years, and the pressure effect of economic development level on environmental quality is higher than the dividend effect. Industrial structure has a positive impact on environmental quality, thereby indicating that optimizing industrial structure is essential in improving environmental quality. This situation benefits from technology diffusion and knowledge spillover brought by the adjustment of industrial structure, thereby enabling enterprises to adopt environmental protection techniques. Moreover, limiting pollution to the range of resource carrying capacity alleviates the negative environmental externality of industrial agglomeration. As expected, the improvement of energy structure and energy efficiency has a relatively positive impact on the entire environment. China’s industrial structure is mainly based on energy, particularly the secondary industry, which that has the highest dependence on energy. The resulting industrial waste gas will have a negative impact on the environment. Hence, improvements in energy structure and energy efficiency will inevitably promote the improvement of environmental quality.

#### 5.2.2 Fixed effect analysis with instrumental variables

When estimating Eq (10), the data is not divided into different regions. The Western, Middle, and Eastern regions should be substituted into the equation to compare the regional differences. If we use pooled regression, the result will not be particularly good, particularly given that some key variables, such as CAED, is not significant. Thereafter, we consider whether the model has fixed effect with regions separately. Owing to the different situation of each province, there may be missing variables that do not change with time. Hence, fixed effect (within estimator) and LSDV method are used for regression analysis, thereby indicating that the fixed effect is evidently better than the pooled regression. Given that the natural evolution is an extremely long period, we assume that there is no time effect but only individual effect, which is denoted by *u*. Hausman test is also conducted to show that the random effect should no longer be considered.

$$\begin{array}{l} LnC_{it}=\alpha +\gamma_{1}LnLAED_{it}+\gamma_{2}LnCAED_{it}+\gamma_{3}LnDED_{it}\\ +\gamma_{4}LnPCGDPit+\gamma_{5}LnIS_{it}+\gamma_{6}LnEF_{it}+\gamma_{7}LnES_{it}+u_{i}+\varepsilon_{it} \end{array}$$ (11)

The preliminary result of Eq (11) is not satisfying because CAED and LAED may be correlated as we discuss on Section 2.2. We attempt to solve it using the instrumental variable method. Through numerous attempts, the fiscal investment of local governments in environmental governance (LFI) has been determined to reflect the government’s effort in environmental governance. The reason is that the local governments’ fiscal investments closely reflect the commands given by the central government. Therefore, LFI is chosen as the instrumental variable of CAED. The specific steps are as follows. (1) The fixed effect model is completed through deviation transformation. (2) CAED is estimated using the instrumental variable. (3) The fixed regression of Eq (11)) is used to obtain the results. Table 5 presents the regression results of Eq (11) for the different regions.

**Table 5:** Regression results of the regions.

	East				Mid				West			
	(1)	(2)	(3)	(4)	(1)	(2)	(3)	(4)	(1)	(2)	(3)	(4)
VARIABLES	lnC	lnC	lnC	lnC	lnC	lnC	lnC	lnC	lnC	lnC	lnC	lnC
lnCAED	-2.068	-1.774*	-1.911*	-1.536**	-0.764**	-0.747**	-0.740**	-0.495***	-1.071	-1.125	-0.533	-0.474
	(1.324)	(0.967)	(1.058)	(0.631)	(0.366)	(0.357)	(0.356)	(0.166)	(0.9)	(0.923)	(0.361)	(0.35)
lnLAED	1.422	1.201*	1.258*	0.874**	0.429*	0.418*	0.411*	0.216*	0.243	0.292	-0.0663	-0.0822
	(0.901)	(0.655)	(0.708)	(0.378)	(0.253)	(0.247)	(0.247)	(0.122)	(0.512)	(0.529)	(0.227)	(0.22)
lnDED	0.0922	0.0778*	0.0877*	0.0669**	0.0521**	0.0513**	0.0507**	0.0380**	0.0518	0.0517	0.0302	0.0259
	(0.059)	(0.0452)	(0.0499)	(0.0336)	(0.0241)	(0.0238)	(0.0238)	(0.0175)	(0.0359)	(0.0363)	(0.0207)	(0.0203)
lnRPGDP	0.46	0.0613	0.359	-0.589**	0.435**	0.415*	0.422*	0.166**	0.904*	0.643	0.23	0.14**
	(1.014)	(0.741)	(0.853)	(0.652)	(0.212)	(0.216)	(0.218)	(0.231)	(0.506)	(0.481)	(0.269)	(0.267)
lnIS		1.446	2.041	1.417		0.179	0.18	-0.00528		1.875*	1.559**	1.534**
		(1.167)	(1.399)	(0.917)		(0.52)	(0.521)	(0.453)		(1.057)	(0.74)	(0.719)
lnEF			0.57	0.334			0.0667	-0.0436			0.331	0.337
			(0.478)	(0.376)			(0.254)	(0.228)			(0.27)	(0.262)
lnES				0.932				0.408				0.305
				(0.644)				(0.286)				(0.223)
Constant	-8.401	-5.263	-11.58	-0.701	-6.763***	-6.684***	-7.070**	-4.059	-13.26**	-12.35*	-7.537**	-7.895***
	(-12.27)	(9.268)	(11.8)	(7.565)	(2.447)	(2.419)	(2.874)	(2.663)	(6.503)	(6.413)	(2.959)	(2.901)
Observations	110	110	110	110	110	110	110	110	110	110	110	110
Number of provincecode	10	10	10	10	10	10	10	10	10	10	10	10

Note: The values in parentheses are standard errors;

*** represents p <0.01,

** represents p <0.05, and

* represents p <0.1.

Given the differences among the Western, Middle, and Eastern regions, Table 5 shows the regression results of the regional difference analysis to further verify the authenticity of the hypothesis. In particular, Table 5 shows that AED of the central government in the three regions remains negatively related to environmental quality, with the Western region having the greatest effect. That is, a 1% increase in the authoritarianism of central government will lead to approximately 1.5%, 0.495%, and 0.474% decline in the environmental qualities of the Eastern, Middle, and Western regions, respectively. The results further verify that H1 is not supported.

Table 5 shows that AED of the local governments in the three regions remains positively related to environmental quality, and the Eastern region continue to have a greater effect than the Middle and Western regions. That is, a 1% strength in the authoritarianism of the central government will cause 0.822%, 0.216%, and 0.874% increases in the environmental qualities of the Western, Middle, and Eastern regions. The results further verify that H2 is supported.

For H3, the positive effects of DED on the environment in the three regions are significant but all coefficients are small. Hence, H3 is supported. People’s appeals for ecological environment convey valuable information and promote environmental improvement through personal participation in environmental protection and effective supervision of governmental actions. However, the effectiveness of DED should be improved.

In terms of the control variables, while the increase of per capita GDP in the Eastern region leads to a decline in environmental quality, an increase of per capita GDP positively affects environmental quality in the Middle and Western regions. It shows that the economic development level in the Middle and Western regions has a higher dividend effect than pressure effect on environmental quality. In other words, economic development and environmental construction are not a pair of contradictions in the Middle and Western regions. It explains that economic development could provide financial and technical support for the ecological environment construction in these two regions. In addition, in terms of industrial structure, the positive effects of industrial structure are significant in the Western and Eastern regions, and the positive effect of industrial structure is significant in the west. Therefore, we suggest that the environmental construction in the Western, Middle, and Eastern regions should focus on the adjustment of industrial structure, improvement of economic development level, and adjustment of industrial structure and ascension of energy efficiency, respectively.

The following is the explanations for the analysis results of the preceding three hypotheses.

First, the contradiction between the authoritarianism of the central and local governments in environmental governance stems from the current environmental governance system in China. The current governance mechanism in China is not a rather than a bottom–up information collection and transmission mechanism, on opposite it is a top–down decision-making and implementation one. Owing to China’s huge governance scale, centralization inevitably leads to contradiction between central decision-making and local policy implementation. This contradiction leads to the fundamental tension between power concentration and effective local governance. The root of the contradiction lies in the idea that the degree of power concentration is at the expense of the effectiveness of local governance. That is, the concentration of power keeps decision-making power and resources away from those levels with substantially accurate information and capabilities in problem solving. By contrast, the enhancement of local governance means that the expansion of local power often leads to (or is interpreted as) deviation from the central government.

Second, empirical analysis shows that the improvement of China’s environmental quality in the past decade is closely related to AED of local governments. The decentralization of local environmental governance has produced various benefits and promoted the improvement of environmental quality in the different regions of China. However, the more centralized resources and decision-making power are, the less effective governance will be. This result is reflected in the lack of initiative of local governments, but the burden on the central government.

Third, the evaluation and assessment systems are only oriented to GDP growth, thereby leading to the fact that the government does not consistently represent the public interest. To maximize the government’s own utility, the government deviates from the goal of maximizing public interest and social welfare. Under this assessment system, the aim to obtain tax and political promotion results in the inevitable tendency of the jurisdiction to accept the pollution industry, thereby forming the counteraction and restriction of AED.

Lastly, the positive effect of DED is less than that of AED of local governments. The core reason is the lack of bottom-up information collection and transmission mechanism in China, and information is filtered or blocked from one governance level to another.

## 6 Conclusions, suggestions, and future directions

### 6.1. Conclusions

We qualitatively and quantitatively explored the effects of AED and DED on environmental quality. The results are as follows. (1) A negative relationship exists between AED of the central government and environmental quality, and this type of negative effect has the highest impact in China’s Western region. (2) A positive relationship exists between AED of local governments and environmental quality, and this type of positive effect also has the highest impact in China’s Eastern region. (3) A positive relationship exists between DED and environmental quality, although the positive effect of DED is weaker than that of AED of local governments throughout China. (4) From the perspective of the relationship between per capita GDP and environmental quality, the pressure effect of economic development on environmental quality is higher than the dividend effect in China. The dividend effect brought by the acceleration of economic development in the Middle and Western regions on environmental quality has begun to be greater than the pressure effect. (5) Industrial structure has a positive impact on environmental quality and the effect is significant in the Western region.

### 6.2 Suggestions

Several policy suggestions are proposed for the preceding conclusions.

First, for AED, we should emphasize the role of local governments in environmental governance. China’s current governance mechanism is a top–down decision-making and implementation mechanism, rather than a bottom–up information collection and transmission mechanism. Such mechanism cannot cope with the huge amount of information of the vast territory of the country and heterogeneous population. The central government attempts to protect itself and filter the information, rather than publicly deal with the scale of information they cannot cope with. However, empirical analysis shows that the government should change its decision-making process, transparency and openness to society in environmental governance, such as decentralizing the power of environmental authorities, particularly for specific environmental affairs limited to local jurisdiction.

Second, for DED, the empirical result has important practical significance for understanding ecological democracy and promoting the improvement of environmental problems. Public participation is the key force to promote environmental protection based on the existence of effective channels for the expression of citizens' interests. The central government, local governments, mass media and non-governmental organizations need to consider how to effectively use this growing power to better guide the public to participate in environmental governance, for ensuring the win-win results of economic growth and environmental improvement. Governments should focus substantially to people’s environmental appeal, which conveys valuable information and promotes the improvement of ecological environment, such as establishing an effective environmental inspection mechanism. Environmental democracy does not disregard government participation and it is not to transfer the solution of environmental problems from the administrative institutions in the hands of the public. In fact, it is to correct and remedy the environmental administrative crisis of governments based on solving problems through democratic means. Its essence is to make administrative institutions considerably democratic and realize the benign interaction between the government and the public by playing the main role of the public.

Third, we should change the evaluation and assessment system that only focuses on GDP growth, and introduce ecological politics into China’s political landscape. Accordingly, green GDP is introduced into the official performance evaluation, including green economic indicators, green security indicators, and green social indicators. Apart from GDP assessment, environmental objectives have become among the most important indicators that local governments should achieve.

Lastly, we suggest that environmental construction in the Western region, which is dominated by coal power, should focus on the optimization, upgrade, and adjustment of the energy structure. Environmental construction in the Middle region should focus on the improvement of economic development level. Environmental construction in the Eastern region should focus on the adjustment of industrial structure and ascension of energy efficiency.

### 6.3 Future directions

The limitation of this research is that such factors as the order of word expression, weight of intensity of the meaning of a word, and effect of word frequency superposition are excluded in the analysis. In addition, the authoritarianism of local government has a spatial attribute because of the proximity of the geographical location and externality of environmental governance. Therefore, the follow-up research should introduce spatial correlation analysis.

## Supporting information

S1 Appendix Key words and word frequency of ecopolitical discourse (Part). (DOCX)

S2 Appendix Index system of the comprehensive level of China’s environmental quality. (DOCX)

S1 Data (XLSX)
